# Preparation of 3D Printing PLGA Scaffold with BMP-9 and P-15 Peptide Hydrogel and Its Application in the Treatment of Bone Defects in Rabbits

**DOI:** 10.1155/2022/1081957

**Published:** 2022-07-31

**Authors:** Xiaomei Wang, Wanjun Chen, Zhe Chen, Yixiu Li, Kai Wu, Yulin Song

**Affiliations:** ^1^Department of Orthopedics, The Second Affiliated Hospital of Nanchang University, Nanchang 330006, China; ^2^Department of Orthopedics, Xiangzhou District People's Hospital, Xiangyang 441000, China; ^3^Department of Pharmacy, The Second Affiliated Hospital of Nanchang University, Nanchang 330006, China

## Abstract

**Objective:**

To prepare a three-dimensional (3D) printing polylactic acid glycolic acid (PLGA) scaffold with bone morphogenetic protein-9 (BMP-9) and P-15 peptide hydrogel and evaluate its application in treating bone defects in rabbits.

**Methods:**

3D printing PLGA scaffolds were formed and scanned by electron microscopy. Their X-ray diffraction (XRD), *in vitro* degradation, and compressive strength were characterized. BMP-9 and P-15 hydrogels were prepared. Flow cytometry was used to detect apoptosis, and an electron microscope was used to evaluate cell adhesion to scaffolds. Alkaline phosphatase (ALP), type 1 collagen (Col-I), osteocalcin (OCN), runt-related transcription factor 2 (RUNX2), and osterix (SP7) were detected by western blotting. MicroCT was used to detect new bone formation, and bone tissue-related protein expressions were determined in the rabbit model with bone defects.

**Results:**

The 3D printing scaffolds were cylindrical, and the inner diameter of the scaffolds was about 1 mm. The bread peak with wide distribution showed that the 3D printing only involved a physical change, which did not change the properties of the materials. The degradation rate of scaffolds was 9.38%, which met the requirements of properties of biological scaffolds. The water absorption of the support was about 9.09%, and the compressive strength was 15.83 N/mm^2^. In the coculture of bone marrow mesenchymal stem cells (BMSCs) with scaffolds, the 2% polypeptide hydrogel showed the most obvious activity in promoting the differentiation of BMSCs. Flow cytometry showed that the 0% and 2% groups did not cause obvious apoptosis compared with the control group. Scaffolds with 2% and 4% polypeptide promoted the expression of ALP, COL-1, OCN, RUNX2, and Sp7 in BMSCs. *In vivo* experiments showed that the expression of ALP, COL-1, OCN, RUNX2, and Sp7 protein in the 2% polypeptide scaffold group increased significantly compared with the model group. MicroCT detection demonstrated that the 2% polypeptide scaffold had good bone repair ability.

**Conclusion:**

The PLGA scaffolds combined with BMP-9 and P-15 peptide hydrogels had good biological and mechanical properties and could repair bone defects in rabbits.

## 1. Introduction

Osteoporosis, bone tumor, and sport-related bone injury contribute to bone defects in different degrees, in which large-scale bone defects seriously affect human health and normal life and could even be the most lethal [1, 2]. The conventional treatment methods for bone defects include autogenous bone transplantation and allogeneic bone transplantation. They both use bone transplantation from other parts of their own or other donors. However, the limited bone resource and exclusion reaction of allogeneic bone transplantation greatly limit bone transplantation's clinical application [3].

Current treatments for bone loss are mainly based on bone transplantation (autologous, allogeneic, or xenogeneic) and biomaterials; however, several factors limit their applications, such as the volume of bone required to adequately treat the traumatic place, lack of vascularization, associated pain, postoperative complications, and other factors that affect the normality of resuming daily activities [4–6]. To help solve such issues, the application of three-dimensional (3D) printing of bone tissue engineering in *ex vivo* models allows the experiments of different materials to assess their interactions with cells, growth factors, and vasculature.

Artificial bone substitute materials have changed from a single chemical bone in the early stage to multicomponent-simulated biological bone materials and have developed into a level close to the natural bone in mechanical and biological functions. With rapid developments in 3D printing technology, its simplicity and accuracy have been improved widely, and 3D printing technology is now commonly used in various fields, such as biomedicine [7]. According to computed tomography (CT), magnetic resonance imaging (MRI), and other imaging data of the injured part of the patient, 3D printing technology can quickly and accurately produce personalized bone tissue engineering scaffolds. CAD technology can also be applied to design any shape according to bone defect requirements and make the 3D scaffolds of any pore structure meet treatment requirements [8, 9].

Polymer materials, with nondegradable and degradable characteristics, are widely used in various aspects of tissue substitute materials due to their excellent properties. Nondegradable materials are stable and can maintain good mechanical properties for a long time, while degradable materials can degrade and be discharged through metabolism or absorbed by the human body [10].

Bone morphogenic protein 9 (BMP-9), also known as growth and differentiation factor 2 (GDF2), is a member of the transforming growth factor *β* (TGF*β*) superfamily. BMP-9 has shown great osteoinductive potential in bone regeneration. P-15 peptide-coated hydroxyapatite promoted bone regeneration in osteoporotic rats. As BMP-9 and P-15 polypeptides have the ability to induce osteoblast proliferation and differentiation through different mechanisms, we prepared chitosan hydrogel embedding both BMP-9 and P-15 polypeptides. Polylactic acid glycolic acid (PLGA) has received considerable attention due to its biocompatibility and biodegradability, and it is among the most used synthetic polymer in the bone regeneration field [11]. Thus, we hypothesized that BMP-9 and P-15 could enhance the bone repair function of the PLGA scaffold, leading to osteoblast-related cells generating new bone.

In this study, we aimed to assess the biological and mechanical properties of BMP-9 and P-15 peptide hydrogels on PLGA scaffolds to repair bone defects in *in vivo* settings. PLGA was used to prepare scaffold material with the assistance of 3D printing technology [12]. The PLGA scaffold containing BMP-9 and P-15 polypeptide hydrogel was prepared, and its influences in rat bone marrow mesenchymal stem cells (BMSCs), as well as in the treatment of bone defects in rabbits, were evaluated.

## 2. Materials and Methods

### 2.1. Experimental Animals

Japanese big ear rabbits were purchased from Nanchang Longping Rabbit Industry Co., Ltd. (license no. SCXK (Gan) 2014–0005). Sprague-Dawley (SD) rats were purchased from Hunan Slake Jingda Experimental Animal Co., Ltd. (license no. SCXK (Xiang) 2016–0002). The animal experiments described in this study were authorized by the Committee of The Second Affiliated Hospital of Nanchang University (no. 202106–261; Nanchang, China) and conducted in compliance with the institutional guidelines for the care and use of animals.

### 2.2. Preparation of 3D Printing PLGA Scaffold

PLGA scaffolds were prepared based upon the melting deposition method as previously described. PLGA raw materials were extruded and deposited by a high-temperature spray nozzle at melting temperature. The scaffolds were formed according to the path controlled by a computer and solidified at room temperature. The 3D graphics of 10 mm (diameter) × 5 mm (height) and 6 mm (diameter) × 8 mm (height) was designed by CAD drawing (Autodesk software, San Francisco, California). The graphics model was imported into 3D-Bioprinter software (Regenovo, Hangzhou, China), and the graphics was stratified. The three-dimensional scaffold was produced using a 3D printer (3D Bio-Architect Pro, Regenovo, Hangzhou, China), placed at room temperature for more than 4 h, and then dried for 12 h in a constant temperature drying oven at 45°C.

### 2.3. Characterization of PLGA Scaffolds

  Pore size analysis: the scaffolds were cut into thin sections and observed under a microscope, and images were taken. After the surface of the scaffolds was sprayed with gold, the pore size and structure were analyzed based on the images using a scanning electron microscope (SEM) (FEI Company, Hillsboro, USA).
  X-ray diffraction (XRD) analysis: an X-ray diffractometer (D8 ADVANCE, Bruker AXS, Karlsruhe, Germany) was used to scan the surface when the scaffold sample was fully dried.
 
*In vitro* degradation: 10 support scaffolds were dried and weighed. Then, the scaffolds were immersed in normal saline at 37°C. One sample was taken out randomly each week. The weight was calculated after drying. The degradation rate was calculated based on the formula: degradation rate (%) = (M0 − M1)/M0 × 100%. M0 and M1 represented the original weight and weight after degradation.
  Determination of water absorption: after weighing the dried scaffold (G), it was placed in 0.9% saline at 37°C for 24 h. Then, the scaffold was taken out and weighted (B). Water absorption was determined using the formula: *W* = ((B − G)/G) × 100%. The average water absorption of three parallel scaffolds was measured.
  Compressive strength analysis: a linear increased pressure was delivered on the cylindrical scaffold at 0.5 mm/min using a microcomputer-controlled electronic universal testing machine (ETM204C, Beijing BIOCOOL, Beijing, China). When the scaffold deformed, the pressure was prohibited.

### 2.4. Preparation of PLGA Scaffold Composite of Polypeptide Hydrogel

Equal amounts of P-15 (Sangon Biotech, Shanghai, China) and BMP-9 (Sangon Biotech, Shanghai, China) were dissolved in 500 *μ*l sterile water, to which 5 ml 2% chitosan acetic acid (0.1 M) was added and mixed. 15 PLGA scaffolds were immersed into the solution for 1 h. After that, 500 *μ*l 100 mg/ml *β*-glycerophosphate and 500 *μ*l 70 mg/ml sodium bicarbonate were added. The mixture was gently shaken at 37°C for 30 h until solidification. The scaffolds were kept at −20°C. 4% polypeptide (4%), 2% polypeptide (2%) and 0% groups were prepared, in which 40 mg P-15 and 40 mg BMP-9, 20 mg P-15 and 20 mg BMP-9, and 0 mg P-15 and 0 mg BMP-9 were included.

### 2.5. Peptide Release from PLGA Scaffold Composite of Peptide Hydrogel

Newborn Sprague Dawley rats were soaked in 75% ethanol for 15–20 min and killed in anoxia. Their tibia and humerus were removed under aseptic condition. Their metaphyseal ends were excised, bone marrow cavity wasexposed and washed thoroughly with 10% complete culture medium, and bone marrow was repeatedly blown out by aseptic syringe so that bone marrow cells were fully separated into single-cell suspension and cultured in Dulbecco's Modified Eagle Medium (DMEM, GIBCO (ThermoFisher, Shanghai, China)) + 20% fetal bovine serum (FBS (ThermoFisher, Shanghai, China)). BMSCs and scaffolds were cocultured. The experiments were divided into 4 groups: a control group (no scaffolds in the orifice plate); a 0% group (scaffolds with hydrogel scaffolds containing 0% peptide); a 2% group (scaffolds with hydrogel scaffolds containing 2% peptide); and a 4% group (scaffolds with hydrogel scaffolds containing 4% peptide). Three days later, the cells were removed from the culture medium, and the scaffolds were detected by SEM.

### 2.6. Measurement of Apoptosis

After washing with PBS, 5 *μ*l Annexin V-fluorescein isothiocyanate (FITC) and propidium iodide (PI) were added and incubated at room temperature in the dark for 10 min, following the manufacturer's instructions. The cells were detected by flow cytometry (NovoCyte 2060R; ACEA Biosciences, Inc., San Diego, CA, USA).

### 2.7. Western Blotting

Total proteins were abstracted from the cells by adding cell lysate solution (28-9425-44, ReadyPrep, GE Healthcare Life Sciences, USA). In brief, the cells with lysate solution were put on ice for 30 min and centrifuged at 4°C for 10 min (10000 ×g), and the supernatant was discarded. The protein concentration was determined using the BCA kit. The protein was denatured and run on 12% sodium dodecyl sulfate-polyacrylamide gel electrophoresis for 1–2 h, followed by wet transferring to nitrocellulose membrane for 30–50 min. The membranes were blocked in 50 defat milk for 2 h at room temperature and incubated with the primary antibodies at 4°C overnight. The primary antibodies included rabbit polyclonal anti-ALP (1 : 1000, PA5-69994, Thermofisher, Shanghai, China), rabbit polyclonal anti-RUNX2 (1 : 200, bs-1134R, Bioss; Shanghai, China), rabbit polyclonal anti-COL-I (1 : 200, bs-0578R, Bioss, Shanghai, China), rabbit polyclonal anti-SP7 (1 : 500, bs-1110R, Bioss, Shanghai, China), and mouse monoclonal anti-OCN (1 : 500, OM266706, OmnimAbs; Shanghai, China). The membranes were then incubated with the secondary antibodies. ECL exposure solution was added to the membrane and exposed to the gel imaging system. The gray values of bands were analyzed by “Quantity One” software.

### 2.8. Animal Model of Bone Injury

The rabbits were prepared after anesthesia, fixed on the operating table on the back and sterilized and covered with a sterile towel, and the right lateral incision of the lower part of the femur (about 3 cm length) was taken. The lateral condyle of the femur and the middle and lower segments of the femur was exposed by incision and subperiosteal stripping. The same side of bone above the articular surface of the lateral condyle of the femur was drilled with a bone drill, then the same side of the bone cortex and internal bone cancellous was chiseled with a bone knife, and the opposite side of the bone cortex remained intact, resulting in a diameter of 7 mm and a depth of about 9 mm. In the same way, two bone defect areas on the left tibia were prepared.

The experiments were divided into the following groups: (1) a control group: without any treatments; a sham group: incision of the model site, separation of periosteum, but no bone damage; (2) a model group: incision of the model site, separation of periosteum, resulting in a 7 mm diameter and 9 mm depth of bone defect; (3) a 0% group: incision of the model site, separation of periosteum, resulting in a 7 mm diameter and 9 mm depth of a bone defect, and PLGA gel scaffold without polypeptide was then implanted into the cavity; (4) a 2% group: incision of the model site, separation of periosteum, resulting in a 7 mm diameter and 9 mm depth of a bone defect, and PLGA gel scaffold containing 2% polypeptides was then implanted into the cavity; and (5) a 4% group: incision of the model site, separation of periosteum, resulting in a 7 mm diameter and 9 mm depth of a bone defect, and PLGA gel scaffold containing 4% peptides was then implanted into the cavity. After the corresponding scaffold materials were implanted, the transplantation area was tightly sutured, and the incision was closed. On the third day after the operation, each animal was given a daily penicillin intramuscular injection to prevent infection in the operation area. The samples were taken on the 8th week after the operation.

### 2.9. MicroCT Detection

The bone samples of rabbits were scanned at 360° by a MicroCT instrument (QuantumGX PerkinElmer Waltham, MA). After a three-dimensional reconstruction of the data, the selected three-dimensional data were analyzed by Analyze12.0.

### 2.10. Statistical Analysis

The data were expressed as mean ± standard deviation by Statistical Package for the Social Sciences v19 (SPSS; IBM, Armonk USA). *T*-test was used to compare the two groups, and single-factor analysis of variance was used to compare multiple groups, followed by the Student–Newman–Keuls *post hoc* test.

## 3. Results

### 3.1. Characterization of PLGA Scaffolds

As shown in Figure 1, the 3D printing scaffold was cylindrical, and the inner diameter was about 1 mm (Figures 1(a)–1(c)). The polycrystalline samples were analyzed by XRD in Figure 1(d). The results of XRD showed a bread peak with wide distribution, indicating the formation of a physical change in the material. The degradation rate for 10 weeks was 9.38%, which indicated that the PLGA scaffold had certain mechanical stability. The water absorption of the scaffold was about 9.09% (Table 1), indicating that it has certain wettability and could adhere to water-soluble substances. Its compressive strength was 15.83 N/mm^2^. The specific characteristics of two peptides of each 2% and 4% scaffolds are shown in Table 1.

### 3.2. Effects of PLGA Scaffold Composite of BMP-9 and P-15 Peptide Hydrogel on Apoptosis of BMSCs

Scanning electron microscopy revealed that the scaffold surfaces adhered with differentiated cells (Figure 2(a)). The scaffolds with the 2% polypeptide were the most obvious to promote cell differentiation, indicating that the scaffolds adhering to polypeptide hydrogel could promote the differentiation of BMSCs cells and were able to attach to scaffolds. There was no difference among the 0% and 2% groups and the control group regarding the apoptosis rate, indicating the scaffolds or scaffolds with 2% BMP-9 and P-15 peptide hydrogel were nontoxic to cells, although the 4% group had a certain effect on apoptosis (Figure 2(b)). Western blotting showed that the expression of ALP, COL-1, OCN, RUNX2, and Sp7 expression in BMSCs cells was enhanced by a single scaffold (0%) and polypeptide scaffold (2% and 4%) (Figure 3).

### 3.3. PLGA Scaffold Composite of BMP-9 and P-15 Peptide Hydrogel Repaired the Bone Defect

As shown in Figure 4(a), the 2% peptide hydrogel group had the most obvious new bone formation (purple-red). The 2% peptide hydrogel scaffold could promote osteoblast-related cells' proliferation and differentiation and induce new bone formation (Figure 4(b)).  Figure 5 shows the expression of ALP, COL-1, OCN, RUNX2, and Sp7 in bone tissue. The results showed that the content of these five proteins in the model group was significantly reduced compared with the control group and sham group, and compared with the model group, the expression of ALP, COL-1, OCN, RUNX2, and Sp7 protein in the 2% polypeptide scaffold group was significantly increased.

## 4. Discussion

3D printing technology includes fused deposition modeling (FDM), stereolithography (SLA), and selective laser sintering (SLS), among others [13]. In this study, the thermoplastic material PLGA was extruded by melting deposition and then moved and piled up according to the designed path under the control of a computer. Finally, the regular morphology, suitable holes and mechanical properties, degradation rate, and biological properties of the scaffold were evaluated. The results showed that the scaffolds had uniform pore size, regular morphology, good biomechanical properties, and degradation ability.

BMP-9 is one of the main factors inducing the osteogenic differentiation of mesenchymal stem cells and plays an important role in the migration of osteoblasts, proliferation of mesenchymal cells, differentiation of cartilage and bone-derived cells, vascular growth, and bone remodeling [14, 15]. P-15 peptide can promote the proliferation and adhesion of fibroblasts and osteoblasts, the secretion of extracellular matrix, and the formation of bone tissue and can also effectively activate and promote the proliferation of mesenchymal stem cells and differentiation into chondrocytes [16]. Therefore, the adhesion of hydrogel to BMP-9 and P-15 can effectively enhance the bone repair function of the PLGA scaffold, promote the proliferation and differentiation of osteoblast-related cells, and generate new bone.

Alkaline phosphatase (ALP) is a specific factor for osteogenesis, which can regulate bone morphogenesis [17]. ALP is a marker enzyme of osteoblasts, which can be used as a specific indicator of osteoblast metabolism [18]. Collagen I (COL-1) is secreted by osteoblasts, which is involved in the development, differentiation, and activity regulation of osteoblasts, and plays an important role in maintaining the biomechanical properties and structural integrity of bone tissue [19]. Osteocalcin (OCN) is a marker of osteoblast differentiation and maturation. The concentration of OCN in blood circulation is closely related to bone metabolism [20]. OCN can attract and combine calcium ions through the negative surface charge of its molecular structure, promote the deposition of calcium, and promote bone formation and calcification of bone [21]. RUNX2 is an osteogenic differentiation-specific transcription factor that can regulate the transcription of many genes [22]. The expression of RUNX2 is important for the differentiation of mesenchymal cells into osteoblasts. The differentiation of osteoblasts in RUNX2 deficient mice is completely inhibited, and periosteal osteogenesis and endochondral osteogenesis do not occur [23]. Sp7 (osteoblast-specific transcription factor osterix) belongs to the SP/xklf family, which is expressed specifically in developing bone tissue and is a necessary transcription factor in osteoblast differentiation and bone formation [24]. According to western blot results, the PLGA scaffold of peptide hydrogel promoted the proliferation and differentiation of rat BMSCs cells and osteogenic induction. Results from the western blot and microCT showed that the PLGA scaffold of peptide hydrogel had a positive effect on bone repair and new bone formation in rabbits.

3D-printed biodegradable PLGA scaffolds provide good attachment and fixation to cells and tissues. The adhesive peptide hydrogels can continuously release P-15 and BMP-9 polypeptide factors with bone induction and differentiation function, stimulate related cells and tissues to secrete COL-1, and upregulate the expression of RUNX2 and many other genes to achieve the purpose of new bone formation and bone repair.

In conclusion, the PLGA scaffolds combined with BMP-9 and P-15 peptide hydrogels demonstrated good biological and mechanical properties and could repair bone defects in rabbits. This new product deserves further clinical study for future application.

## Figures and Tables

**Figure 1:** Characterization of PLGA scaffolds. (a) Images observed under light microscope; (b) structure observed under scanning electron microscope; (c) surface polypeptide hydrogel observed under scanning electron microscope; (d) XRD analysis; (e) degradation rate; (f) peptide release rate.

**Figure 2:** Effects of PLGA scaffold composite of BMP-9 and P-15 peptide hydrogel on apoptosis of BMSCs. (a) SEM characterization; (b) flow cytometry detection of apoptosis. Compared with the control group, ^*∗*^*P* < 0.05.

**Figure 3:** PLGA scaffold composite of BMP-9 and P-15 peptide hydrogel promoted ALP, COL-1, OCN, Runx2, and Sp7 protein expression in BMSCs. Compared with the control group, ^*∗*^*P* < 0.05.

**Figure 4:** PLGA scaffold composite of BMP-9 and P-15 peptide hydrogel repaired the bone defect. (a) Animal modeling process. (b) MicroCT test (blue, scaffold; pink, new bone).

**Figure 5:** PLGA scaffold composite of BMP-9 and P-15 peptide hydrogel promoted ALP, COL-1, OCN, RUNX2, and Sp7 expression in bone tissue. Compared with the control group, ^*∗*^*P* < 0.05. Compared with the model group, ^#^*P* < 0.05.

**Table 1:** Characterization of PLGA scaffolds.

Test items	Results (*n* = 3)
Water absorption	9.09 ± 0.65%
Compressive strength	15.83 ± 0.42 N/mm^2^
Peptide loading capacity (2% peptide)	0.227 mg P-15; 0.227 mg BMP-9 (per scaffold)
Peptide loading capacity (4% peptide)	0.462 mg P-15; 0.462 mg BMP-9 (per scaffold)

## Data Availability

The data used to support the findings of this study are available from the corresponding author upon request.

## Abbreviations

3D: Three-dimensional
PLGA: Polylactic acid glycolic acid
BMP-9: Bone morphogenetic protein-9
XRD: X-ray diffraction
ALP: Alkaline phosphatase
Col-I: Type 1 collagen
OCN: Osteocalcin
RUNX2: Runt-related transcription factor 2
SP7: Osterix
BMSCs: Bone marrow mesenchymal stem cells
MRI: Magnetic resonance imaging
CT: Computed tomography
TGF*β*: Transforming growth factor *β*
SD: Sprague-Dawley
SEM: Scanning electron microscope
DMEM: Dulbecco's Modified Eagle Medium
FBS: Fetal bovine serum
FITC: Fluorescein isothiocyanate
PI: Propidium iodide
SPSS: Statistical Package for the Social Sciences
FDM: Fused deposition modeling
SLA: Stereolithography
SLS: Selective laser sintering
ALP: Alkaline phosphatase.
